RETRACTED

# An Orthopedic Auxiliary Diagnosis System Based on Image Recognition Technology

**DOI:** 10.1155/2021/4644392

**Published:** 2021-11-22

**Authors:** Yang Guo, Chen Chen

**Affiliations:** First Affiliated Hospital of Xiamen University, Xiamen 361000, China

## Abstract

There are many kinds of orthopedic diseases with complex professional background, and it is easy to miss diagnosis and misdiagnosis. The computer-aided diagnosis system of orthopedic diseases based on the key technology of medical image processing can locate and display the lesion location area by visualization, measuring and providing disease diagnosis indexes. It is of great significance to assist orthopedic doctors to diagnose orthopedic diseases from the perspective of visual vision and quantitative indicators, which can improve the diagnosis rate and accuracy of orthopedic diseases, reduce the pain of patients, and shorten the treatment time of diseases. To solve the problem of possible spatial inconsistency of medical images of orthopedic diseases, we propose an image registration method based on volume feature point selection and Powell. Through the linear search strategy of golden section method and Powell algorithm optimization, the best spatial transformation parameters are found, which maximizes the normalized mutual information between images to be registered, thus ensuring the consistency of two-dimensional spatial positions. According to the proposed algorithm, a computer-aided diagnosis system of orthopedic diseases is developed and designed independently. The system consists of five modules, which can complete many functions such as medical image input and output, algorithm processing, and effect display. The experimental results show that the system developed in this paper has good results in cartilage tissue segmentation, bone and urate agglomeration segmentation, urate agglomeration artifact removal, two-dimensional and three-dimensional image registration, and visualization. The system can be applied to clinical gout and cartilage defect diagnosis and evaluation, providing sufficient basis to assist doctors in making diagnosis decisions.

## 1. Introduction

Due to the improvement of living standards, the number of patients with orthopedic diseases is rising day by day. The number of patients with lumbar spondylosis in China alone reaches 15.2% of the total population, which has become another major disease endangering human health. There are many kinds of orthopedic diseases. Some symptoms are similar and may occur at the same time. Traditional diagnosis methods of orthopedic diseases lack sufficient information to assist doctors in diagnosis, which easily leads to missed diagnosis and misdiagnosis, delays patients' treatment, and may even cause medical accidents. According to statistics, the misdiagnosis rate based on medical images can reach 10%–30%. Computer-aided diagnosis technology is called the “third eye” of doctors, which can not only greatly improve the diagnosis speed of doctors, but also improve the accuracy of diagnosis results. Therefore, it is of great practical significance to use computer-aided diagnosis technology to diagnose orthopedic diseases [1].

RETRACTED

Computer-aided diagnosis technology includes computer science, medicine, mathematics, graphics, and other multidisciplinary knowledge, covering numbers, images, and three-dimensional models [2]. Its realization depends on medical image and its processing technology. Image modes such as computed tomography, microscopic computed tomography, and high-power microscope imaging can record various pieces of information. Combined with medical image processing technologies such as image segmentation, registration, and visualization, useful information can be visually presented by integrating index values, two-dimensional images, and three-dimensional models. This changes the previous way that doctors make diagnosis through experience or spatial imagination with the help of two-dimensional images. The method provides many scientific bases for diagnosis and makes computer-aided diagnosis technology be more widely used [3].

Because of intellectual property rights and bundled sales, these systems are expensive and cannot be open source. On the other hand, these systems meet the diagnostic needs of most cases, but they cannot be applied to the diagnosis of orthopedic diseases in specific or complex scenarios. Based on these factors, in order to solve the specific complex orthopedic disease aided diagnosis, we must design our own computer-aided diagnosis system. Therefore, this paper combines the computer-aided diagnosis system based on medical image processing with the diagnosis process of orthopedic diseases. A computer-aided diagnosis system for orthopedic diseases is designed and developed. The auxiliary diagnosis and evaluation of common orthopedic diseases gout and cartilage defect are realized. The technical problems of medical image processing, such as image segmentation, image registration, and visualization, are studied and analyzed. Using dual-energy CT, segmentation, visualization, and other algorithms, the urate crystal area and three-dimensional model of gout are detected and displayed, and the total volume of urate crystal is measured. The cartilage defect area and three-dimensional model containing internal structure in the image to be diagnosed are detected and displayed by using the cartilage image to be diagnosed. The complete cartilage template contains internal structure of cartilage in the data bone bank and algorithms such as segmentation, registration, and visualization. It provides sufficient basis for doctors to diagnose and evaluate the degree of gout and cartilage defect and is also of great significance for subsequent gout treatment and cartilage tissue surgical repair [4].

RETRACTED

With the continuous development of science and technology, the innovative technology of medical images is also closely related to the progress of science and technology. We designed a two-dimensional image object measurement system including system package and software package, which can be used together with imaging, processing, and displayed devices. This system mainly shoots images and measures the size and orientation of objects to locate surgical tools and structures in images during surgery [5]. This system provides a template method for drawing and displaying information and data values of visible objects in images. Although ultrasound examination has been completely popularized, it is widely used in the examination of various patients. But its value has not been fully utilized. In view of this phenomenon, we searched the database and found that bedside ultrasound diagnosis and treatment is helpful to orthopedic surgeons. It is also sensitive to the evaluation of partial and total rotator cuff tears in orthopedic clinic. Compared with guided injection, ultrasound can improve the accuracy of injection and may be helpful to doctors' diagnosis [6]. Intelligent sensors have been widely used in communication, industry, and other industries. Orthoses play an important role in medical field, which can not only protect joints, but also relieve pain. The combination of orthoses and sensors enables doctors to master patients' parameters, get more reliable results, and help them understand their illness. We propose the fact that wireless intelligent sensors and field programmable gate array (FPGA) [7] can mainly monitor pressure and reduce internal tissue necrosis. Experiments show that they can be effectively used in orthopedic field.

The structure of this paper is as follows: Section 2 introduces the proposed image registration method and the method testing results; Section 3 presents the developed diagnosis system and the system testing results; Section 4 concludes this paper and gives future research directions.

## 2. Image Registration Method Based on Volume Feature Point Selection and Powell in Auxiliary Diagnosis of Orthopedic Diseases

Image registration can align the spatial positions between images [8]. Combined with image fusion, multidata information can be presented on the same image to assist diagnosis. Image registration needs two objects, floating image and reference image, and it is actually a process of mapping floating image to reference image one by one. The purpose is to make the pixels in reference image correspond to each other in floating image, and the overall spatial position of the image is consistent [9]. Image registration is very important in the process of computer-aided diagnosis of orthopedic diseases, which can be used for auxiliary diagnosis of cartilage defects and tracking the effect before and after gout treatment [10]. Osteoarthritis is a disease caused by cartilage degeneration at joints. Osteophyte, cartilage sclerosis, and shortening of joint space are its internal symptoms. X-ray scanning of synovial fluid is a common method to diagnose osteoarthritis, but the early symptoms of osteoarthritis are not obvious, and it is easy to miss diagnosis and misdiagnosis. In order to solve this problem, many scholars have carried out research on auxiliary diagnosis of osteoarthritis. Fracture is one of the most common orthopedic diseases. External force or long-term strain is the main cause of fracture. General fracture is easy to diagnose because of its obvious external characteristics, but incomplete fracture, deep fracture, intra-articular fracture, and tiny fracture are often difficult to detect clinically, which may lead to missed diagnosis. At present, the auxiliary diagnosis of fracture is mainly to find out the characteristics that can describe bone.

RETRACTED

### 2.1. Image Registration Algorithm Based on Powell

The complete cartilage template image contains the information of internal structure areas such as hyaline cartilage layer, calcified cartilage layer, and subchondral bone layer, which needs doctors to take pictures under high-power microscope through histological staining sections. In this way, some artificial or uncertain factors may cause deformation such as translation or deflection between slices [11]. Therefore, in order to reshape the spatial relationship between slices, a Powell-based image registration algorithm is proposed. The algorithm takes one of the complete cartilage template image sequences as the reference image, the other as the floating image, and takes the normalized mutual information value between the reference image and the floating image as the similarity measure, which is maximized by optimizing iteration to achieve the best registration effect, thus completing the construction of the complete cartilage template [12].

In this paper, complete color cartilage slices obtained under the same high-power microscope are used as images to be registered, and the size and physical pixel spacing of each slice image are kept consistent to realize image data normalization. To avoid the influence of sundries and noise in the image background, firstly, the image is preprocessed by cartilage segmentation. Only the key regions of interest that need to be registered in spatial position are reserved. This part of the work has been completed in the previous chapter; then, one image is selected as the reference image, and the other images are used as floating images. The floating image and the reference image are registered by Powell algorithm, including linear search, transformation interpolation, and calculation of normalized mutual information. Then, the best parameters obtained from registration are used to transform the floating image to complete the whole registration process. The specific algorithm flow chart is shown in Figure 1.

RETRACTED

### 2.2. Image Space Transformation and Interpolation

As can be seen from Figure 1, image transformation is the key part of image registration algorithm. Common image transformation methods include rigid body transformation, affine transformation, projection transformation, and nonlinear transformation [13]. In this paper, orthopedic diseases are mainly studied, so rigid body transformation is adopted. The characteristic of rigid body transformation is that the distance between any two pixels in the image remains unchanged after transformation, so it is mainly rotation and translation transformation. The process of image rigid body transformation involves the original point (*x*, *y*), the transformed point (*x*_1_, *y*_1_), the translation distance *m* along the horizontal direction, the translation distance *n* along the vertical direction, and the rotation angle *σ* around the center point (*x*_*c*_, *y*_*c*_) of the image. The realization of rotation transformation in rigid body transformation depends on the rotation matrix, as shown in

(1) $$\begin{array}{c} \left[\begin{array}{c} x_{1}-x_{c}\\ y_{1}-y_{c} \end{array}\right]=\left[\begin{array}{cc} \cos\;\sigma & -\sin\;\sigma \\ \sin\;\sigma & \cos\;\sigma \end{array}\right]\left[\begin{array}{c} x-x_{c}\\ y-y_{c} \end{array}\right]. \end{array}$$

The realization of translation transformation depends on translation matrix, as shown in

(2) $$\begin{array}{c} \left[\begin{array}{c} x_{1}-x_{c}\\ y_{1}-y_{c}\\ 1 \end{array}\right]=\left[\begin{array}{ccc} 1 & 0 & m\\ 0 & 1 & n\\ 0 & 0 & 1 \end{array}\right]\left[\begin{array}{c} \begin{array}{c} x-x_{c}\\ y-y_{c} \end{array}\\ 1 \end{array}\right]. \end{array}$$

The sequence of the two operations also has an impact on the calculation. See the following equation for the calculation method of translation before rotation:

(3) $$\begin{array}{c} \left[\begin{array}{c} x_{1}-x_{c}\\ y_{1}-y_{c}\\ 1 \end{array}\right]=\left[\begin{array}{ccc} \cos\;\sigma & -\sin\;\sigma & m\;\cos\;\sigma -n\;\sin\;\sigma \\ \sin\;\sigma & \cos\;\sigma & m\;\sin\;\sigma +n\;\cos\;\sigma \\ 0 & 0 & 1 \end{array}\right]\left[\begin{array}{c} \begin{array}{c} x-x_{c}\\ y-y_{c} \end{array}\\ 1 \end{array}\right]. \end{array}$$

See the following equation for the calculation equation of first rotation and then translation:

(4) $$\begin{array}{c} \left[\begin{array}{c} x_{1}-x_{c}\\ y_{1}-y_{c}\\ 1 \end{array}\right]=\left[\begin{array}{ccc} \cos\;\sigma & -\sin\;\sigma & m\\ \sin\;\sigma & \cos\;\sigma & n\\ 0 & 0 & 1 \end{array}\right]\left[\begin{array}{c} \begin{array}{c} x-x_{c}\\ y-y_{c} \end{array}\\ 1 \end{array}\right]. \end{array}$$

It can be seen that the calculation of (4) is relatively simple compared with (3), so (4) is used in the transformation process of two-dimensional registration of complete cartilage template images.

RETRACTED

Image interpolation is carried out simultaneously with image transformation, which is used to solve the problem of obtaining the gray value of pixels after image transformation. The digital image only stores the gray information of pixels at integer coordinates and rarely keeps integers after the coordinate positions of image pixels are transformed. Therefore, it is inevitable to interpolate the image to keep the image information basically consistent before and after transformation [14]. The effect of image interpolation is related to the implementation of specific algorithm. The higher the accuracy of the algorithm, the clearer the interpolated image and the more complex the calculation [15]. In this paper, bilinear interpolation and partial volume interpolation are mainly used in the two-dimensional registration algorithm of complete cartilage template images.

Bilinear interpolation is the most commonly used interpolation method [16], which can keep the texture detailed information in the image basically unchanged with the transformation. Nonlinear interpolation is realized by performing three times of one-dimensional linear interpolation in horizontal and vertical directions, as shown in Figure 2(a). When the transformed pixel *q*(*x*_*q*_, *y*_*q*_) falls in a noninteger region, the gray value of the pixel is only related to the gray value of four adjacent integer pixels (*x*_*q*_, *y*_*q*_), (*x*_*q*_+1, *y*_*q*_), (*x*_*q*_, *y*_*q*_+1), and (*x*_*q*_+1, *y*_*q*_+1)

(5) $$\begin{array}{c} f\left(x_{q},y_{p}\right)=f\left(x_{p},y_{p}\right)+u\left[f\left(x_{p}+1,y_{p}\right)-f\left(x_{p},y_{p}\right)\right], \end{array}$$

(6) $$\begin{array}{c} f\left(x_{q},y_{p}+1\right)=f\left(x_{p},y_{p}+1\right)+u\left[f\left(x_{p}+1,y_{p}+1\right)-f\left(x_{p},y_{p}+1\right)\right], \end{array}$$

(7) $$\begin{array}{c} f\left(x_{q},y_{q}\right)=f\left(x_{q},y_{p}\right)+v\left[f\left(x_{q},y_{p}+1\right)-f\left(x_{q},y_{p}\right)\right]. \end{array}$$

Formulas (5)–(7) are formula conversions of positions, and their positional relationships can be seen in Figure 2.

RETRACTED

Different from bilinear interpolation method, PV interpolation uses the gray joint histogram information of two images to be registered in the complete cartilage template and updates the joint histogram directly without gray interpolation, so that new pixels do not need to be generated, and the error caused by rounding in gray interpolation will not be brought, as shown in Figure 2(b). Image registration based on mutual information completely depends on the histogram of gray distribution, so PV interpolation fits this kind of image registration perfectly, which can make the calculation of mutual information more accurate and help to search the best registration parameters. In this paper, PV interpolation [17, 18] is used to calculate the normalized mutual information between complete cartilage images. The calculation process of PV interpolation is as follows:

(8) $$\begin{array}{c} h_{fr}\left(f\left(p_{i}\right),r\left(x\right)\right)+=w_{i},\;i=1,2,3,4,\\ w_{1}=\left(1-u\right)\left(1-v\right),\\ w_{2}=u\left(1-v\right),\\ w_{3}=\left(1-u\right)v,\\ w_{4}=uv, \end{array}$$

where *r* (*x*) denotes the whole cartilage floating image, *f* (*x*) denotes the whole cartilage reference image, and *h*_*fr*_(*f*(*p*_*i*_), *r*(*x*)) is the gray statistic of the gray histogram between them.

### 2.3. Target Decision Function Based on Normalized Mutual Information

Mutual information is a common method to measure the correlation between two objects in informatics theory. The application of mutual information in medical image registration can measure the similarity between images, and there is no need for gray relationship between images. Therefore, this paper takes the normalized mutual information as the standard function of Powell algorithm on the basis of mutual information calculation [19, 20].

Mutual information is used to measure the statistical correlation between the gray values of corresponding pixels in image registration, so the calculation of mutual information is related to probability statistics and needs to be expressed by entropy. Entropy is a quantity describing the uncertainty of an image. The more complex and chaotic the image is, the greater the entropy is. For the image to be registered, the calculation of entropy depends on the probability density of gray distribution. The probability that the gray value of pixels in the image is *i* can be expressed by *P*_*f*_(*i*)=(*C*(*i*)/*M*), *M* is the total number of pixels, and *C* (*i*) is the number of pixels with gray value *I*. The joint density distribution between the gray value *i* in the reference image and its corresponding floating image gray value *j* can be expressed as *P*_*fr*_(*i*, *j*)=(*C*(*i*, *j*)/*N*), where *C*(*i*, *j*) represents the number of pixel pairs with gray level *i* in the reference image and gray level *j* in the floating image, and *N* represents the number of all pixel pairs. In this way, according to the definition of entropy, the information entropy *H* (*F* (*i*)) and *H* (*R* (*J*)) of reference image *F* (*i*) and floating image *R* (*J*) as well as their joint information entropy *H* (*F* (*i*), *R* (*J*)) and conditional information entropy *H*(*f*(*i*)*|r*(*j*)) or *H*(*r*(*j*)*|f*(*i*)) can be obtained, as shown in the following formula:

(9) $$\begin{array}{c} H\left(f\left(i\right)\right)=-\sum_{i}P\left(i\right)\log\;P\left(i\right),\\ H\left(r\left(j\right)\right)=-\sum_{j}P\left(j\right)\log\;P\left(j\right),\\ H\left(f\left(i\right),r\left(j\right)\right)=-\sum_{i,j}P\left(i,j\right)\log\;P\left(i,j\right),\\ H\left(f\left(i\right)|r\left(j\right)\right)=-\sum_{i,j}P\left(i,j\right)\log\;P\left(i|j\right),\\ H\left(r\left(j\right)|f\left(i\right)\right)=-\sum_{i,j}P\left(i,j\right)\log\;P\left(j|i\right). \end{array}$$

Mutual information represents the reduction of uncertainty of floating image *R* (*J*) when reference image *F* (*I*) is known. The greater the mutual information, the smaller the uncertainty of *R* (*J*), indicating that images *F* (*I*) and *R* (*J*) are more similar. See the following equation for specific calculation:

(10) $$\begin{array}{c} I\left(f\left(i\right),r\left(j\right)\right)=H\left(f\left(i\right)\right)-H\left(f\left(i\right)|r\left(j\right)\right)\\ =H\left(f\left(i\right)\right)+H\left(r\left(j\right)\right)-H\left(f\left(i\right),r\left(j\right)\right). \end{array}$$

The specific relationship between mutual information and various entropies is shown in Figure 3.

RETRACTED

According to the probability density distribution, mutual information can also be expressed by

(11) $$\begin{array}{c} I\left(f\left(i\right),r\left(j\right)\right)=\sum_{i,j}P\left(i,j\right)\log\frac{P\left(i|j\right)}{P\left(i\right)}. \end{array}$$

In addition, mutual information also has the following important properties:

1. Symmetry: *I* (*f* (*i*), *r* (*j*)) = *I* (*r* (*j*), *f* (*i*)); this indicates that the information of the image *r* (*j*) extracted from the image *f* (*i*) is the same as the information of the image *f* (*i*) extracted from the image *r* (*j*).
2. Nonnegativity: *I* (*f* (*i*), *r* (*j*)) ≥ 0; the greater the similarity of the images *f* (*i*), *r* (*j*), the greater the mutual information. When *f* (*i*), *r* (*j*) are independent of each other, the mutual information is 0.
3. Extreme value: *I* (*f* (*i*), *r* (*j*)) ≤ *H* (*f* (*i*)) and *I* (*f* (*i*), *r* (*j*)) ≤ *H* (*r* (*j*)).
4. Convex functionality: the second derivative of *I* (*f* (*i*), *r* (*j*)) is always nonnegative.

In order to reduce the complexity of image registration, the reference image is often not transformed, but only the floating image is transformed. When the floating image transformation does not lose useful information, the registration effect based on mutual information is often very good, but when there is loss, the overlapping area with the reference image becomes smaller, and the registration will fall into local extremum, which makes the effect very bad. To solve this problem, entropy correlation coefficient is introduced, and the expression is shown in

(12) $$\begin{array}{c} \text{ECC}\left(f\left(i\right),r\left(j\right)\right)=\frac{I\left(f\left(i\right),r\left(j\right)\right)}{H\left(f\left(i\right)+H\left(r\left(j\right)\right.\right)}. \end{array}$$

Then, in order to further simplify the operation, normalized mutual information is introduced, which is expressed by

(13) $$\begin{array}{c} \text{NMI}\left(f\left(i\right),r\left(j\right)\right)=\frac{H\left(f\left(i\right)\right)+H\left(r\left(j\right)\right)}{H\left(f\left(i\right),r\left(j\right)\right)}. \end{array}$$

From the expressions (11)–(13), it can be known that ECC and NMI change the relationship between edge entropy and joint entropy from addition and subtraction to ratio relationship, which greatly improves the accuracy of image registration.

In addition, on the basis of mutual information properties, normalized mutual information also has the property of boundedness; that is, 1 ≤ NMI ≤ 2. When images are independent of each other, NMI is 1, and when images are completely identical, NMI is 2. In order to improve the registration accuracy and simplify the calculation, the normalized mutual information expression is used as the objective function of two-dimensional registration of complete cartilage templates, and the spatial position alignment between complete cartilage images is realized by maximizing the objective function value through iterative changes of translation and rotation angles.

### 2.4. Parameter Search Algorithm Based on Golden Section Method

Parameter search algorithm is needed to find the optimal translation and rotation parameters, and the quality of the search algorithm is related to the search speed and the accuracy of the final registration. Powell algorithm is a direct search algorithm, which has high requirements for the search direction. It must require that the search direction is linearly independent; otherwise it is easy to fall into the local optimal solution. The improved Powell algorithm solves this problem well. Powell algorithm has high computational efficiency and fast convergence speed. It can quickly and accurately find the optimal parameters and complete high-precision image registration.

RETRACTED

One-dimensional search algorithm can not only solve the optimal solution problem in one dimension, but also has a good effect on realizing multidimensional search. Common one-dimensional search algorithms include interval elimination method, golden section method [21], Newton method, and parabola method. The golden section method is established on the basis of interval elimination method to improve convergence speed, and it is faster than Newton method because it does not need derivative operation like Newton method. Although the golden section method is slower than the parabola method, the accuracy and reliability of the results are higher than the latter. In this paper, we need to consider the search speed and the accuracy and reliability of the results, so in Powell algorithm the golden section method is used to search the spatial transformation parameters of the complete cartilage floating image.

The golden section method is a one-dimensional search algorithm [22]. In the multidimensional case, one parameter is guaranteed to be optimal first, then the next one-dimensional optimal search is carried out, and finally all the best parameters are searched. The steps of searching for the optimal parameters by golden section method are as follows:

1. Set the initial search interval [*a*, *b*] and the accuracy requirement *e* and then calculate the intermediate points *c*, *d*: *c* = *a* + 0.382 (*b* − *a*), *d* = *a* + 0.618 (*b* − *a*), and calculate the function values *f* (*c*) and *f* (*d*) according to the objective function *f* (*x*).
2. Judge that *b* − *a* < *e*; stop the search if it is true; at this time, the objective function obtains the extreme value *f* ((*b* + *a*)/2) at (*b* + *a*)/2; if it is not true, judge the size of *f* (*c*) and *f* (*d*); if *f* (*c*) > *f* (*d*), go to step 3; if *f* (*c*) ≤ *f* (*d*), go to step 4.
3. Set *f* (*c*) = *f* (*d*), *a* = *c*, *c* = *d*, and *d* = *a* + 0.618 (*b* − *a*), calculate *f* (*d*), and return to step 2.
4. Set *f* (*d*) = *f* (*C*), *b* = *d*, *d* = *c*, and *c* = *a* + 0.382 (*b* − *a*), calculate *f* (*c*), and return to step 2.

RETRACTED

### 2.5. Image Registration Effect Verification

In order to verify the effectiveness of the image registration algorithm used in this paper in aligning the internal spatial position of the complete cartilage template, several groups of experiments were designed from the perspective of accuracy and time efficiency [23]. The idea of experimental design is to randomly select 5 cartilage images from 54 complete cartilage images, then, they are rotated and translated with the same set *X*, *Y*, and angle offset values, and the set parameter values are recorded. Finally, the image before transformation is used as reference image and the image after transformation is used as floating image. Using this algorithm, we can get a set of *X*, *Y*, and angle parameter values. By comparing these two sets of values, we can verify the two-dimensional registration effect. The closer the parameter value is to the opposite number of the set offset value, the better the registration effect is. The experimental results are shown in Table 1.

It can be seen from Table 1 that the difference between *X* and *Y* offsets of registration results is between −0.4 and +0.1, the difference between angle offset values is between −0.1 and 0.1, the average time required for each registration operation is 4.38 s, and the average normalized mutual information value (NMI) is 1.762, which shows that the image similarity after registration is high, which fully shows that the image registration algorithm introduced in this section is effective from the perspective of quantitative indicators.

In addition, it can also verify the effect of the image registration algorithm from the most direct visual perspective. Two-dimensional registration of complete cartilage images is carried out by using the image registration algorithm in this paper, there are 54 complete cartilage images, and the image size is 544^*∗*^818. The contrast effect before and after registration of two randomly selected images is shown in Figure 4. Figures 4(a) and 4(c) show the relative position relationship between the reference image and the floating image before two-dimensional registration, and Figures 4(b) and 4(d) show the relative position relationship between the reference image and the floating image after two-dimensional registration using this algorithm. After visual comparison, it can be easily known that the spatial position relationship within the complete cartilage template is basically the same after image registration by this algorithm, so the complete cartilage template sequence can be constructed by this method for subsequent registration.

RETRACTED

## 3. Design of Computer-Aided Diagnosis System for Orthopedic Diseases

As an effective tool, computer-aided diagnosis plays an increasingly important role in the actual diagnosis and treatment of orthopedic diseases [24]. In order to facilitate for doctors operating or showing the effect of algorithm realization, the realization of computer-aided diagnosis technology usually needs the help of software system. The system must be able to read and analyze medical images of various modes, and at the same time it can realize various algorithms with concise structure and powerful functions. In addition, due to the complexity of various diseases, in order to facilitate the customization of functions, the system should also be easy to modify and expand.

At present, the computer-aided diagnosis system, which is widely used in the field of orthopedic diagnosis, generally has the characteristics of broad functions and mature design, which can realize routine orthopedic disease diagnosis, but it is not effective for complex or specific orthopedic diseases, and it is basically not open source, so it is impossible to design orthopedic disease aided diagnosis with its source code. Based on these factors, this paper independently designed a computer-aided diagnosis system for orthopedic diseases [25] and realized the auxiliary diagnosis functions of gout and cartilage defect with the help of this system.

### 3.1. System Modules

The computer-aided diagnosis system of orthopedic diseases designed in this paper mainly realizes the functions of gout aided diagnosis and cartilage defect aided diagnosis. The system has perfect functions and simple operation and can provide orthopedic doctors with many pieces of information such as two-dimensional and three-dimensional images and index values for diagnosis. Hardware of this system design and development environment: HP Z800 Workstation, CPU Intel Xeon (R) X5690, graphics card Nvidia Quadro 5800 4G; software: Win10 64-bit operating system, VS2020, MFC, OpenGL; programming language: C++.

Modular development of software system can not only make software structure clear and content concise, but also be easy to modify, expand, and increase functions. Using modular idea, the system is divided into five modules: image data reading and analysis, image data preprocessing, key algorithm realization of gout auxiliary diagnosis, key algorithm realization of cartilage defect auxiliary diagnosis, and data display and output. The overall framework is shown in Figure 5.

Image data reading and analysis module mainly includes dual-energy CT sequence, timing reference image sequence, floating image sequence image reading, and analysis. Its function is to convert DICOM, Raw, and other format images into easy-to-display BMP format. Image data preprocessing module can be subdivided into image smoothing and image enhancement. Image smoothing includes median filtering, mean filtering, and Gaussian filtering, and image enhancement includes histogram equalization and window level and width transformation. The function of this module is mainly to create conditions for the realization of subsequent algorithms. The key algorithm implementation module of gout aided diagnosis is responsible for realizing computer-aided gout diagnosis function, including bone and urate crystal region segmentation algorithm, bone and urate crystal region three-dimensional reconstruction algorithm, and urate crystal artifact removal algorithm. The key algorithm implementation module of cartilage defect aided diagnosis is responsible for realizing the computer-aided cartilage defect diagnosis function, including cartilage segmentation algorithm, two-dimensional registration algorithm of complete cartilage template image in digital bone bank, three-dimensional registration algorithm of cartilage image to be diagnosed and complete cartilage template, and three-dimensional reconstruction algorithm of cartilage and defect position. The data display and output module is responsible for displaying and outputting data images. It includes index data display, image display, image data output, and rapid prototyping file output. The output of image data is to derive two-dimensional BMP image, and the output of rapid prototyping file is to generate and derive three-dimensional .stl, .iges, and .obj format files, which can be directly used for 3D printing. Each module complements each other and cooperates together, which constitutes a complete computer-aided diagnosis system for orthopedic diseases.

RETRACTED

### 3.2. Implementation Flow of Gout Auxiliary Diagnosis Function Module

The realization process of gout auxiliary diagnosis is roughly divided into four parts: dual-energy CT sequence reading, bone and urate crystal region segmentation, three-dimensional reconstruction, and urate crystal artifact removal, as shown in Figure 6.

Among them, the reading of dual-energy CT sequence mainly involves the analysis of DICOM picture format, bone and urate crystal region segmentation using the third section of Chapter 2 based on threshold segmentation region growth and logistic regression bone and urate crystal region segmentation algorithm, three-dimensional reconstruction using the improved MC three-dimensional reconstruction algorithm based on multiregion labels in the second section of Chapter 4 that can reconstruct the three-dimensional model of bone region and the three-dimensional model of urate crystal region at the same time. The urate crystallization artifact removal algorithm based on three-dimensional volume segmentation and region labeling is used in the fourth section of Chapter 2. Each part of the process is interrelated and cooperates with each other to assist doctors in gout diagnosis from two angles of three-dimensional visualization and quantitative analysis of indicators in Figure 6.

### 3.3. Actual Case Verification of Gout Auxiliary Diagnosis Function

In order to verify the accuracy and effectiveness of the gout diagnosis function of this system, this section uses actual cases to assist doctors in gout diagnosis on the computer-aided diagnosis system of orthopedic diseases in this paper. The patients with gout had swollen dorsum of foot with pain. Dual-energy CT was performed on Siemens CT machine, and CT sequences at 80 kV and 140 kV were obtained. There is a problem with the units here, and the correct ones should be row = 512, column = 512, pieces number = 315, pixel spacing = 0.486 mm, and interlayer spacing = 1.0 mm in Figure 7.

According to the quality of the imported image, you can choose whether to preprocess the image or not. The image quality of this case is clear, so the preprocessing operation steps are omitted. In order to realize the segmentation algorithm of bone and urate crystal region, it is necessary to select “urate crystal segmentation adjustment panel,” in which the threshold of threshold segmentation is set, and the segmentation operation will be carried out. The red region represents urate crystal and the blue region represents bone. Then, provide three-dimensional diagnostic information for obtaining three-dimensional model and obtain three-dimensional model in three-dimensional view window. Green represents urate crystallization area, red represents corroded bone area, and white represents bone area. Because there are some artifacts near toes in this case, therefore, it is necessary to use urate artifact removal algorithm to remove false positive areas; through the “Artifact Removal” menu, the accurate urate crystallization area and 3D model can be obtained by selecting the appropriate removal method. As shown in Figure 8, an enlarged 3D model is shown with urate crystallization artifact removed, and Figure 8(b) is the final 3D model after urate crystallization artifact removed.

In addition, on the “3D Model Info” display panel, select the “Update” button command to obtain information such as Bone Triangular Pieces NUM, MSU Triangular Pieces NUM, MSU Ratio, and MSU VOL.

RETRACTED

In this case, it is obvious that there are large urate crystal areas by two-dimensional and three-dimensional visualization methods, and the total volume of urate crystals also indicates that the content of urate crystals is very high, so the doctor made a diagnosis decision that he suffered from severe gout and needed subsequent resection treatment.

### 3.4. Realization Flow of Functional Module for Auxiliary Diagnosis of Cartilage Defect

Combined with the previous algorithm research, the realization process of cartilage defect auxiliary diagnosis is divided into four parts: reference image processing, complete cartilage template construction, 3D image registration, and 3D image fusion, as shown in Figure 9.

Among them, reference image processing involves the introduction and analysis of cartilage images to be diagnosed, preprocessing and cartilage segmentation, and cartilage segmentation uses cartilage segmentation methods based on threshold and morphological operations; the construction of complete cartilage template includes import and analysis of complete cartilage image, preprocessing, cartilage segmentation, and two-dimensional image registration. Cartilage segmentation adopts cartilage segmentation method based on edge and morphological operation, and two-dimensional image registration is realized by two-dimensional image registration algorithm based on Powell. Three-dimensional image registration can align the spatial position between the cartilage image to be diagnosed and the complete cartilage template; three-dimensional image fusion adopts the method of obtaining cartilage defect area and three-dimensional model. In addition, the registration and fusion of three-dimensional images need to use the improved MC three-dimensional reconstruction algorithm based on multiregion labels for three-dimensional reconstruction. Through this series of processing, the cartilage defect area and three-dimensional model including internal structure in the cartilage image to be diagnosed can be obtained, which can assist doctors to diagnose and evaluate the degree of cartilage defect.

### 3.5. Actual Case Verification of Auxiliary Diagnosis Function of Cartilage Defect

In order to verify the accuracy and effectiveness of this system, this section uses actual cases to assist doctors in the diagnosis of cartilage defects on this computer-aided diagnosis system. The diagnostic object was knee cartilage, and the format was micro-CT sequence generated by high-resolution micro-CT system, with the size of 500*∗*500*∗*500, pixel spacing = 0.04 mm, and interlayer spacing = 0.04 mm. The complete cartilage template is taken from the digital bone bank, which contains RGB color images of cartilage tissue slices of various parts obtained by doctors under Nikon DS-Ri2 high-power microscope and standardized data format. The normal and intact knee cartilage template was derived from the digitized bone bank. The size of the template was 818*∗*544*∗*54, pixel spacing = 0.025 mm, and the interlayer spacing was 0.025 mm.

RETRACTED

The cartilage image to be diagnosed can be imported by the command “Open MatchImg1” under the “File” menu, and the complete cartilage template image can be imported by the command “OpenMatchImg2.” After importing, the image display effect is as shown in 10. The left side is the reference image of cartilage to be diagnosed, and the right side is the complete cartilage image. Information such as image size, quantity, layer spacing, and pixel spacing can be obtained in the rightmost image information panel. In the process of importing cartilage, MATLAB engine has been used for cartilage segmentation of the image to be diagnosed, and the resolution of each direction has been increased by 10 times in order to clearly display the three-dimensional model in Figure 10.

Because the spatial position slice directions of the reference image and the floating image in this case are inconsistent, it is necessary to realize the spatial transformation of the reference image of cartilage to be diagnosed by the “RefImg Transformation” command in the “Soft Restructuring” menu, so as to ensure that the slice directions of the two images are basically consistent. The transformed results are shown in Figure 11, and it can be seen that the slice directions of the two image sequences are consistent.

In order to normalize the three-dimensional data field, it is necessary to use the “Data Normalization” command to make the layer spacing and pixel spacing of the reference image and the floating image consistent. As shown in Figure 12, not only the layer spacing and pixel spacing of the two sequences are unified to 0.25 mm, but also the size of each image slice is unified to 800*∗*800.

In order to obtain the reference 3D model and floating 3D model, it is necessary to use the “3D Reconstruction” command to run the improved MC 3D reconstruction algorithm with multiregion labels. As shown in Figure 13, gray indicates the reference 3D model of cartilage to be diagnosed, and yellow indicates the floating 3D model of complete cartilage.

In order to obtain the cartilage defect area and three-dimensional model in the cartilage image to be diagnosed, the command “Get SofiROI” is needed. As shown in Figure 14, the reference image and fusion image show the cartilage defect area, and the three-dimensional model of the cartilage defect site is displayed in the three-dimensional view.

RETRACTED

In this case, the cartilage defect area including internal structure and three-dimensional model in the cartilage image to be diagnosed can be visually displayed by the two-dimensional and three-dimensional visualization methods of this system. Doctors can clearly observe that there is cartilage defect in this case and there is a large subchondral bone layer area in the defective cartilage tissue, which indicates that the defect is large and it is difficult to repair and heal by itself. Therefore, doctors make a diagnosis decision that the cartilage defect exists in this case and needs subsequent cartilage repair surgery.

## 4. Conclusion

The purpose of this paper is to apply computer diagnosis technology to the diagnosis of orthopedic diseases; a computer-aided diagnosis system for orthopedic diseases was built independently. Firstly, the modules and interfaces are introduced. According to the modular design, the platform is divided into five modules: image data reading and analysis, image data preprocessing, key algorithm realization of gout auxiliary diagnosis, key algorithm realization of cartilage defect auxiliary diagnosis, and data display and output. The interface is used to operate and display image data. After that, the functions of gout aided diagnosis and cartilage defect diagnosis are realized on the computer-aided diagnosis system of orthopedic diseases by using the algorithm operation in the previous chapter. Through the process overview and actual case verification, it is proved that the system can provide useful information such as quantitative indicators and two-dimensional and three-dimensional visualization. This can accurately and effectively assist doctors in diagnosis and has positive significance to improve the efficiency and accuracy of gout diagnosis and cartilage defect diagnosis.

## Figures and Tables

**Figure 1:** Flow chart of two-dimensional image registration algorithm based on Powell.

**Figure 2:** Schematic diagram of common two-dimensional interpolation algorithm. (a) Schematic diagram of bilinear interpolation. (b) Schematic diagram of partial volume interpolation.

**Figure 3:** Relationship diagram of mutual information entropy $\begin{array}{ccc} H\left(f\left(i\right),r\left(j\right)\right) & H\left(r\left(j\right)\right) & H\left(r\left(j\right)|f\left(i\right)\right) \end{array}$.

**Figure 4:** Comparison renderings before and after registration of actual floating images. (a) Preregistration example I. (b) Example I after registration. (c) Preregistration example II. (d) Preregistration example II.

**Figure 5:** Overall frame diagram of computer-aided diagnosis system for orthopedic diseases.

RETRACTED

**Figure 6:** Implementation flow chart of gout auxiliary diagnosis function module.

**Figure 7:** Introducing and parsing dual-energy CT sequences.

**Figure 8:** Three-dimensional model images before and after removing false positives. (a) Before removing urate crystallization artifacts. (b) After removing the urate crystallization artifacts.

**Figure 9:** Realization flow of functional module for auxiliary diagnosis of cartilage defect.

**Figure 10:** Importing reference image and floating image.

**Figure 11:** Spatial transformation of reference image.

**Figure 12:** Normalization processing of three-dimensional volume data field.

**Figure 13:** Dimensional image registration.

**Figure 14:** Defect cartilage tissue area and three-dimensional model acquisition.

**Table 1:** Two-dimensional registration algorithm test experimental data table.

Experimental group	Data category	*X* offset (mm)	*Y* offset (mm)	Angle offset (°)	Time consumption (s)	NMI value
Test 1	Set offset value	10	0	0	4.67	1.672
	Registration parameter value	−9.6881	−0.2428	−0.0619		
Test 2	Set offset value	0	10	0	3.12	1.853
	Registration parameter value	0.0536	−10.0484	−0.0213		
Test 3	Set offset value	0	0	20	3.46	1.587
	Registration parameter value	0.1248	−0.1682	−19.9770		
Test 4	Set offset value	10	10	0	5.13	1.784
	Registration parameter value	−9.9952	−9.8156	−0.0023		
Test 5	Set offset value	10	0	20	5.32	1.752
	Registration parameter value	−9.8972	0.1384	−19.9622		

## Data Availability

The experimental data used to support the findings of this study are available from the corresponding author upon request.
